The article "lncRNA HOTAIR Inhibition by Regulating HMGB1/ROS/NF-κB Signal Pathway Promotes the Recovery of Spinal Cord Function" was retracted in 2023. Reasons: signs of a paper mill; compromised peer review; unreliable results or conclusions.

# lncRNA HOTAIR Inhibition by Regulating HMGB1/ROS/NF-*κ*B Signal Pathway Promotes the Recovery of Spinal Cord Function

**DOI:** 10.1155/2022/4955982

**Published:** 2022-06-28

**Authors:** Zhe Wang, Ruchao Long, Zhihua Yang, Chunzhi Feng

**Affiliations:** Department of Orthopaedics, Affiliated Xiaoshan Hospital, Hangzhou Normal University, Zhejiang Hangzhou 311200, China

## Abstract

Spinal cord ischemia-reperfusion injury (SCII) is one of the most serious complications of clinical aortic aneurysm and vascular malformation surgery. Long noncoding RNA (lncRNA) is involved in the progression of SCII, whereas long noncoding RNA HOX transcript antisense RNA (lncRNA HOTAIR) is unclear in SCII. This study is aimed at confirming the role and related mechanism of HOTAIR in SCII. Later on, a model of SCII was established by clamping the aortic arch for 14 minutes. RNA expression of HOTAIR was detected via qRT-PCR at 12 h, 24 h, 36 h, and 48 h after SCII. The Tarlov scoring system and TUNEL assay were used to evaluate neurological function and neuronal apoptosis. Oxidative stress factor levels were assessed according to the instructions of the kit. Inflammatory cytokines were assessed by ELISA. Western blot was used to detect levels of p65, p-p65, I-*κ*B*α*, and p-I-*κ*B*α*. We found HOTAIR was raised in SCII rats. si-HOTAIR was able to reverse SCII-induced oxidative stress in SCII rats. The HMGB1 expression was upregulated in SCII tissues and negatively correlated with HOTAIR. HMGB1 was able to partially reverse si-HOTAIR inhibition of oxidative stress, inflammatory injury, and neuronal cell apoptosis in SCII. In addition, the ROS/NF-*κ*B signaling pathway is involved in HOTAIR/HMGB1 regulation of SCII. In a word, HOTAIR inhibition is able to inhibit oxidative stress, inflammatory injury, and neuronal apoptosis in SCII through downregulation of the high mobility group protein B1(HMGB1), which is achieved by inhibiting the ROS/NF-*κ*B signaling pathway. The HOTAIR/HMGB1/ROS/NF-*κ*B molecular pathway may be a new mechanism for the treatment of SCII.

## 1. Introduction

Spinal cord ischemia-reperfusion injury (SCII) is a serious injury to the central nervous system. The pathophysiological process after SCII is very complex, mainly including free radical damage, calcium channel opening, lipid peroxidation, and apoptosis, which often causes very serious damage to nerve cells and becomes an obstacle to later recovery [1, 2]. The incidence of acute and delayed paraplegia due to SCII ranges from 3% to 18%, placing a huge emotional and financial burden on the patient's family and society [3, 4]. Despite current improvements in surgical techniques and perioperative management, SCII is still impossible to fully predict and prevent. There is less and less scope for reducing the duration of ischemia through improved surgical techniques and their associated ancillary technologies [5, 6]. Therefore, it is necessary to find new ways of protecting the spinal cord.

Long noncoding RNA (lncRNA) is a class of RNA molecules greater than 200 nt in length that function at the transcriptional, posttranscriptional, and epigenetic levels, but do not encode proteins themselves, and is involved in physiological functions in a variety of ways [7, 8]. It has an important regulatory role in the development of the central nervous system and in the pathology of neurodegenerative diseases and is specifically highly expressed in the central nervous system [9, 10]. HOX transcript antisense RNA (HOTAIR) is an lncRNA obtained by transcription of the HOXC motif, which is first reported to regulate the expression of the HOXD gene [11]. Follow-up studies have found that HOTAIR is also involved in different human diseases such as cancer, heart diseases, and rheumatoid arthritis, and it has been shown that HOTAIR plays an important role in the nervous system [12–14]. For SCII, it is unclear whether HOTAIR is involved in the regulation of this pathophysiology.

High mobility group box 1 (HMGB1) is a class of evolutionarily highly conserved nonhistone DNA-binding proteins that are widely found in eukaryotic cells. HMGB1 in the nucleus plays a role in stabilizing nucleosomes, regulating gene transcription, and participating in DNA recombination, repair, and replication [15]. Previous studies have focused on its intranuclear function. It has been found that HMGB1 can be released extracellularly and mediate inflammatory responses. The inflammatory role of extracellular HMGB1 has attracted extensive attention both nationally and internationally [16]. Follow-up studies have shown that HMGB1, which enters the extracellular medium, can act as an important inflammatory mediator in the development of various diseases, such as sepsis, arthritis, and ischemia-reperfusion injury [17–19]. In SCII, HMGB1 can promote oxidative stress and inflammatory damage [20]. The role of HOTAIR in regulating HMGB1 in SCII is unclear. The ROS/NF-*κ*B pathway is involved in the progression of a variety of diseases. These include cancer, cardiovascular disease, inflammatory damage, and oxidative stress damage [21, 22]. Previous studies suggest that isoquercetin prevents oxidative stress and neuronal apoptosis in cerebral ischemia-reperfusion injury by inhibiting the ROS/NF-*κ*B pathway [23].

In view of the above research basis, this experiment was intended to explore the effect of HOTAIR regulation of HMGB1/ROS/NF-*κ*B on SCII by establishing a rat model of SCII and provide a reference for clinical prevention and treatment of SCII. We found that HOTAIR was significantly increased in SCII rats. HMGB1 expression was upregulated in SCII tissues and negatively correlated with HOTAIR. HMGB1 was able to partially reverse si-HOTAIR inhibition of oxidative stress, inflammatory injury, and neuronal cell apoptosis in SCII. In addition, the ROS/NF-*κ*B signaling pathway is involved in the HOTAIR/HMGB1 regulation of SCII.

## 2. Materials and Methods

### 2.1. Animals

50 adult male Wistar rats of SPF grade, weighing 250 ± 10 g, were provided by the Benxi Experimental Animal Centre, China Medical University. The rats were housed for one week in an adaptive free range. The rats were randomly divided into 5 groups of 10 rats each. The rats underwent the same cannulation and the same surgical and anesthetic procedures as the other groups but without blocking the thoracic aorta; group SCII (12 h, 24 h, 36 h, and 48 h): the rats were clamped at the arch of the thoracic aorta between the left common carotid artery and the left subclavian artery for 14 min and then opened to cause ischemia/reperfusion injury to the spinal cord; the tissues were taken at different time points of 12 h, 24 h, 36 h, and 48 h of ischemia/reperfusion.

### 2.2. Establishment of Animal Surgical Models

The rats were anesthetized with 4% sodium pentobarbital (50 mg/kg) by intraperitoneal injection, a temperature probe was placed in the rectum, and the core temperature was maintained at 37.0 ± 0.5°C with an electric blanket. A PE50 catheter was first inserted into the left common carotid artery and then into the caudal artery, and the rat's proximal mean arterial blood pressure (PMAP) and distal mean arterial pressure (DMAP) were monitored with a monitor. The skin of the neck was exposed, disinfected, and prepared; a median cervical incision was made; the trachea was fully exposed and then tracheally intubated and connected to a small animal ventilator for assisted ventilation (tidal volume 2 ml/100 g, respiratory rate 80-100 breaths/min, respiratory ratio = 1 : 1). The chest was elevated in the right lateral position, and a curved incision of approximately 4 cm in length was made below the left scapula in the direction of the intercostal space. Carefully dissect the intercostal muscle between the 2nd and 3rd ribs to reveal the apical or upper lobe of the lung; protect the apical lung with dry gauze to reveal the pulmonary veins and pericardium. The aortic arch between the left subclavian artery and the left common carotid artery was clamped with an arterial clip and reopened 14 minutes after clamping. The thoracic cavity was hemostatic, a venipuncture needle was left in place, an airtight environment was prepared with a 10–20 ml syringe, adequate suction was applied, the chest was closed layer by layer, the skin was sutured, and penicillin was injected intramuscularly to prevent infection. After good respiratory recovery, the tracheal tube was removed, the skin of the neck was sutured, and the rats were returned to the cage for rearing. After the thoracic aortic block, the rats were monitored with a Doppler blood flow monitor for a 90% decrease in blood flow in the caudal artery, confirming that the block was reliable, and the ischemic effect was confirmed.

### 2.3. Collection of Materials

After anesthesia, spinal cord tissues from L2 to L5 segments were removed, fixed in 4% paraformaldehyde at 4°C and paraffin embedded for immunohistochemical staining. After satisfactory anesthesia, the spinal cord was quickly removed from the L2 to L5 segments and stored in EP tubes at -80°C for Western blot and qRT-PCR.

### 2.4. Intrathecal Injection

After anesthesia, the back of each rat was flexed, and a 25 *μ*l microinjector was inserted between the L4 and L6 segments of the subarachnoid space. Loss of resistance on needle insertion, the presence of a tail-flick, and the presence of cerebrospinal fluid in the needle were three signs of correct position. The timing and dose of plasmid sheath injection was determined by preexperimentation and qRT-PCR to verify the results. We performed intrathecal injections at 24-hour intervals 3 days before surgery, and rats with normal motor function were moulded. Lipofectamine 3000 was used to transfect the plasmid at a final drug concentration of 2.5 *μ*g/*μ*l. si-HOTAIR and si-NC.HMGB1 were purchased from Nanjing Kingsway Biologicals.

### 2.5. qRT-PCR

Tissue RNA was extracted by the TRIzol method. After removal of genomic DNA in a 10 *μ*l reaction system, reverse transcription was performed in a 20 *μ*l reaction system to obtain cDNA. Reaction conditions are as follows: prereaction at 37°C for 15 min and reaction at 85°C for 5 s. The cDNA samples obtained after reverse transcription were diluted in a 10-fold gradient, 20 *μ*l Master Mix reaction solution was added to the PCR tubes, and GAPDH was used as the control. The CaMKIV gene was detected via qRT-PCR using the ABI7500 qRT-PCR system. After the reaction, the target gene amplification curves were analyzed using the ABI7500 analysis software, and the corresponding standard curves were plotted. The expression level of the CaMKIV gene in the spinal cord of the SCII group was measured using GAPDH as the reference gene, and the sham-operated group was used as the calibration sample to compare the expression difference of the SCII group relative to the sham-operated group and analyzed using the 2^-△△Ct^ method. HOTAIR: F: 5′-CAGTGGGGAACTCTGACTCG-3′, R: 5′-GTGCCTGGTGCTCTCTTACC-3′; HMGB1: F: 5′-ATCCCAATGCACCCAAGAGGCCT-3′, R: 5′-TTCGCAACATCACCAATGGACAGG-3′; GAPDH: F: 5′-GCAGTCATCCTTCTCTCAGT-3′, R: 5′-GTATGCAGTAGCTTGTTACTT-3′.

### 2.6. Tarlov Scores

Two observers assessed the neuromotor function of the hind limbs of the rats using the Tarlov scale, which was described as follows: 0, no lower limb motor function; 1, poor lower limb motor function with weak detectable movement; 2, some joint movement in the lower limbs but no standing; 3, standing but no normal walking; 4, normal.

### 2.7. TUNEL

Tissue sections were routinely dewaxed, ethanolized to rehydration step by step, rinsed in distilled water, pepsin digested for 60 minutes, and rinsed in running water to abort the reaction. Tissue sections were rinsed with buffer, and then, 50 *μ*l of labelling solution was added dropwise to cover the sections, rinsed twice with PBS, placed in an endogenous enzyme blocker, rinsed for 2 minutes with PBS, spotted with HRP-avidin in a wet box, washed twice with PBS and DABH202 for 10 minutes, rinsed under running water, dehydrated routinely, and sealed with gum. The reagents were provided by the Beijing Zhongshan Jinqiao Company; please refer to the kit instructions for details. Apoptotic cells were identified as positive cells with brownish granules in the nucleus under the microscope. To observe apoptotic cells under a light microscope, 18 high magnification fields (×400) were randomly selected in the distribution area of apoptotic cells in each group (one section from each of 10 rats in each group, 3 fields were taken from each section), and the number of apoptotic cells was counted.

### 2.8. Spinal Cord Tissue Biochemical Indicators

A 1-11.5 cm piece of spinal cord tissue was removed from the centre of the lumbar expansion (L4-6) of the rat spinal cord, added to saline prechilled to 4°C according to 1 : 9, and homogenised, and then, the supernatant was taken, divided, and frozen. The brain tissues were then homogenised, and the supernatants were separated and frozen. The contents of SOD, MDA, NO, GSH, and GST were determined via spectrophotometric methods according to the instructions of the kit.

### 2.9. ELISA

The levels of IL-6, TNF-*α*, and IL-1*β* were measured via enzyme-linked immunosorbent assay (ELISA) in rat spinal cord tissues of each group.

### 2.10. Detection of ROS

ROS was detected by DCFH-DA staining. DCFH-DA itself did not emit fluorescence and can enter the cell through the cell membrane. DCFH-DA was hydrolyzed to DCFH by lipase in the cell. Nonfluorescent DCFH will be oxidized to fluorescent DCF when encountering reactive oxygen species. The specific steps were as follows: prepared DCFH-DA working solution, made a drop, moved the tissue to be tested into the incubator at 37°C and 5% CO_2_ for 15 min, washed it for 10 times, and observed it with fluorescence microscope.

### 2.11. Western Blot

Took the spinal cord segment with a length of about 5 mm, added protein lysate, determined the protein content with ultraviolet spectrophotometer, took the same amount of protein sample, separated the protein via SDS-PAGE electrophoresis, transferred the protein band to PVDF membrane via the semidry method, and blocked it with 1% BSA for 1 h; p65 (1 : 1000), p-p65 (1 : 1000), I-*κ*B*α* (1 : 1000), p-I-*κ*B*α* (1 : 1000), and GAPDH (1 : 2000) were put and cultivated under 4°C all night. HRP-labelled secondary antibodies (1 : 2500) were cultivated at room temperature for 1 hour. The band was analyzed via ImageJ, and the gray level of the targeted protein was expressed as the proportion of the gray value of the targeted protein band to the gray value of the GAPDH band. All antibodies were bought from Abcam (UK).

### 2.12. Statistical Research

This study used the SPSS 20.0 statistical software for analysis. Statistical data were shown as average ± SD, one-way ANOVA and *t* test were utilized to make a comparison between groups, and the LSD experiment was utilized for two-way comparison. *P* ≤ 0.05 meant the difference was statistically significant.

## 3. Results

### 3.1. HOTAIR Was Upregulated in SCII Rats

Analysis of PCR results from sham group, 12 h group, 24 h group, 36 h group, and 48 h group after SCII suggested that the expression of HOTAIR was significantly higher at 24 h after SCII (*P* < 0.05, Figure 1(a)). The lower limb function of SCII rats were assessed at the time point of 24 h of SCII. The results showed that the Tarlov score was significantly lower in the SCII group, compared to the sham group (*P* < 0.05, Figure 1(b)). TUNEL results showed that the number of apoptotic neuronal cells was significantly higher in the SCII 24 group compared to the sham group (*P* < 0.05, Figure 1(c)). Furthermore, the oxidative stress factor MDA was significantly increased in the SCII group, while SOD was decreased (*P* < 0.05, Figures 1(d) and 1(e)). ELISA showed an increase in IL-6 and IL-1*β* at 24 h in SCII, compared to sham (*P* < 0.05, Figures 1(f) and 1(g)).

### 3.2. HOTAIR Downregulation Alleviated Oxidative Stress in SCII Rats

Later on, siRNA targeting HOTAIR (si-HOTAIR) and negative control (si-NC) were injected intrathecally into SCII rats to assess the effect of HOTAIR inhibition on oxidative stress in SCII rats. qRT-PCR results showed that HOTAIR was absent in the SCII+si-HOTAIR group compared to the SCII group (*P* < 0.05, Figure 2(a)). The Tarlov score was significantly higher in the si-HOTAIR group, compared to the SCII group (*P* < 0.05, Figure 2(b)). Assessment of oxidative stress factor levels indicated that SCII significantly upregulated MDA and NO and downregulated SOD, GSH, and GST levels (*P* < 0.05, Figures 2(c)–2(g)). However, si-HOTAIR was able to reverse the SCII-induced changes in oxidative stress factor levels in SCII rats.

### 3.3. HOTAIR Downregulation Alleviated Inflammatory Damage in SCII Rats

Subsequently, the effect of HOTAIR inhibition on inflammatory injury in SCII rats was assessed. ELISA results showed that levels of inflammatory cytokines IL-6, TNF-*α*, and IL-1*β* were expanded and levels of IL-4 and IL-10 were absent in the SCII+si-HOTAIR group compared to the sham group. However, IL-6, TNF-*α*, and IL-1*β* levels were suppressed and IL-4 and IL-10 levels were expanded in the SCII+si-HOTAIR group compared to the SCII group (*P* < 0.05, Figures 3(a)–3(e)). Similarly, qRT-PCR showed the same trend for the above inflammatory cytokines at the mRNA level (*P* < 0.05, Figures 3(f)–3(j)).

### 3.4. HOTAIR Was Positively Correlated with HMGB1

HMGB1 has been shown to promote inflammatory injury and apoptosis in SCII [20]. qRT-PCR results confirmed that HMGB1 levels were expanded in the SCII group compared to the sham group (*P* < 0.05, Figure 4(a)). However, HMGB1 levels were inhibited by si-HOTAIR in SCII (*P* < 0.05, Figure 4(b)). The effects of si-HOTAIR/HMGB1 on oxidative stress, inflammatory injury, and apoptosis in SCII rats were assessed by intrathecal injection of siRNA against HOTAIR (si-HOTAIR) and HMGB1 overexpression plasmid. The results showed that HMGB1 intervention increased MDA and downregulated SOD compared with the SCII+si-HOTAIR group (*P* < 0.05, Figures 4(c) and 4(d)). Similarly, ELISA showed that HMGB1 increased IL-6 and IL-1*β* in si-HOTAIR-interfered SCII rats (*P* < 0.05, Figures 4(e) and 4(f)). Furthermore, TUNEL showed that HMGB1 intervention was able to increase the number of apoptotic neuronal cells, compared to the SCII+si-HOTAIR group (*P* < 0.05, Figure 4(g)).

### 3.5. HOTAIR Inhibition Promoted Recovery of Spinal Cord Function in Rats with SIC by Modulating the HMGB1/ROS/NF-*κ*B Signaling Pathway

Finally, the involvement of the ROS/NF-*κ*B signaling pathway in the regulation of SCII by HOTAIR/HMGB1 was assessed. The ROS inhibitor NAC was injected intraperitoneally into SCII rats. ROS staining showed that si-HOTAIR downregulated the relative expression levels of ROS in SCII rats. HMGB1 partially reversed the effect of si-HOTAIR; however, NAC was able to downregulate the levels of ROS in SCII rats (*P* < 0.05, Figure 5(a)). Western blot results showed that si-HOTAIR downregulated the relative expression levels of p65/p-p65 and I-*κ*B*α*/p-I-*κ*B*α* in SCII rats. HMGB1 partially reversed the effect of si-HOTAIR; however, NAC was able to downregulate p65/p-p65 and I-*κ*B*α*/p-I-*κ*B*α* in SCII rats (*P* < 0.05, Figure 5(b)).

## 4. Discussion

Spinal cord ischemia/reperfusion injury is a condition in which the spinal cord tissue has been ischemic for a certain period of time, and after the ischemic factors have been removed and blood perfusion has been restored, the spinal cord neurological function does not improve but is instead aggravated by the original ischemic injury, and even irreversible spinal cord neuronal death occurs [24]. SCII is the leading cause of postoperative paraplegia after spinal surgery, thoracoabdominal aortic aneurysm, and other surgical procedures, which not only seriously impairs the patient's physical and mental health but also places a burden on family and society. As perioperative SCII has a certain degree of predictability, it is not only feasible but also significant to take active measures to prevent and treat SCII at an early stage [25]. With the increasing sophistication of the department and interventional procedures, there is limited scope for further surgical reduction of SCII, and therefore, new approaches need to be explored to mitigate SCII.

lncRNAs are specifically and highly expressed in the central nervous system and have important regulatory roles, such as participating in the development of the central nervous system and in the pathology of neurodegenerative-related diseases [26, 27]. The pathophysiology of ischemia-reperfusion injury in the spinal cord, an important component of the central nervous system, has similarities to that of brain tissue. For instance, downregulation of lncRNA GAS5 inhibited apoptosis and inflammatory responses after spinal cord ischemia-reperfusion in rats [28]. Qiao et al. demonstrated that lncRNA MALAT1 was neuroprotective in a rat model of spinal cord ischemia-reperfusion injury through miR-204 regulation [29].

It is unclear whether HOTAIR is involved in the pathophysiology of SCII and plays a corresponding role. In the present study, the modelled rats, all of which showed lower limb motor dysfunction, demonstrated successful SCII modelling. Similarly, changes in HOTAIR expression occurred 12 h after moulding, with HOTAIR significantly increased in SCII rats and a significant increase in expression at 24 h. This suggests that HOTAIR may promote SCII progression.

Oxidative stress injury plays an important role in SCII. Large amounts of oxygen free radicals are generated during spinal cord ischemia [30, 31]. These oxygen radicals can cause changes in the lipid microenvironment such as membrane receptors, membrane proteases, and ion channels, which can cause impaired cell metabolism, cellular edema, and ultimately apoptosis. Malondialdehyde (MDA) is produced as a result of lipid peroxidation reactions on cell membranes, and MDA production is used as strong evidence of postreperfusion injury [32, 33]. In the current study, we found that SCII caused an upregulation of the oxidative stress factor MDA and a downregulation of SOD. This suggests that SCII caused oxidative stress damage. Furthermore, HOTAIR knockdown was able to downregulate MDA and NO and upregulate SOD, GST, and GSH, suggesting that HOTAIR could alleviate SCII-induced oxidative stress injury.

The inflammatory response plays an important role in SCII. The mechanism of the ischemia-induced inflammatory response is complex and results from the interaction of cytokines, inflammatory chemokines, adhesion factors, free radicals, and destructive enzymes such as cyclooxygenase (COX-1), inducible NO synthase, and proteases [34]. The inflammatory response occurs not only in severe acute SCII but also in the period following Wallerian degeneration of the spinal white matter. Studies have shown increased levels of plasma inflammatory mediators, including cytokines (IL-6, IL-1*β*, TNF-*α*, IL-4, IL-8, and IL-10) and soluble IL-2 receptors, in patients with advanced SCII, and these findings reinforce the role of the inflammatory response in secondary damage to the spinal cord [35]. In the current study, SCII caused upregulation of the inflammatory factors IL-6 and IL-1*β*, suggesting that inflammatory damage is involved in SCII. On the other hand, si-HOTAIR intervention was able to downregulate IL-6, IL-1*β*, and TNF-*α* and upregulate IL-4 and IL-10, suggesting that HOTAIR is able to alleviate SCII-induced inflammatory damage.

HMGB1 has been shown to be involved in inflammatory and oxidative stress and apoptosis through multiple signaling pathways including WNT, Keap1/Nrf2/ARE, and PI3K/AKT [36–38]. Furthermore, previous studies have confirmed the role of the ROS/NF-*κ*B pathway in activating HMGB1 in TDI-induced inflammatory injury [39]. In the current study, we found a significant expansion of HMGB1 in SCII. And HMGB1 was able to partially reverse the inhibitory effects of HOTAIR on oxidative stress, inflammatory damage, and apoptosis. In addition, Western blot showed activation of the ROS/NF-*κ*B pathway in the SCII rat model. This suggests that HOTAIR in SCII acts through HMGB1/ROS/NF-*κ*B. However, there are certain shortcomings in this study. Firstly, we investigated the role and mechanism of HOTAIR in SCII by constructing a rat model of SCII. However, human and cellular experiments need to be further validated. In addition, HMGB1 is involved in inflammation and oxidative stress injury through the regulation of multiple signaling pathways, and whether HOTAIR can regulate other downstream pathways needs to be further explored. In conclusion, HOTAIR inhibition is able to inhibit oxidative stress, inflammatory injury, and neuronal apoptosis in SCII through downregulation of HMGB1, which is achieved by inhibiting the ROS/NF-*κ*B signaling pathway. The HOTAIR/HMGB1/ROS/NF-*κ*B molecular pathway may be a new mechanism for the treatment of SCII.

## Figures and Tables

**Figure 1:** HOTAIR was upregulated in SCII rats. (a) qRT-PCR for HOTAIR expression. (b) Lower limb function score. (c) TUNEL assay for apoptosis. (d, e) MDA and SOD levels were measured according to the kit instructions. (f, g) ELISA for IL-6 and IL-1*β* levels. ^∗∗∗^*P* < 0.001, compared with sham group.

**Figure 2:** HOTAIR downregulation alleviated oxidative stress in SCII rats. (a) qRT-PCR assay for HOTAIR expression. (b) Lower limb function score. (c–g) MDA, SOD, NO, GSH, and GST levels were measured according to the kit instructions. ^∗∗∗^*P* < 0.001, compared with the sham group; ^###^*P* < 0.001, compared with the SCII+si-NC group.

**Figure 3:** HOTAIR downregulation alleviated inflammatory damage in SCII rats. (a–e) ELISA for IL-6, TNF-*α*, IL-1*β*, IL-4, and IL-10 levels. (f–j) qRT-PCR for IL-6,TNF-*α*, IL-1*β*, IL-4, and IL-10 mRNA levels. ^∗∗∗^*P* < 0.001, compared with the sham group; ^###^*P* < 0.001, compared with the SCII+si-NC group.

**Figure 4:** HOTAIR was positively correlated with HMGB1. (a, b) qRT-PCR assay for HMGB1 expression. (c, d) MDA and SOD levels were measured according to the kit instructions. (e, f) ELISA for IL-6 and IL-1*β* levels. (g) TUNEL assay for apoptosis. ^∗∗∗^*P* < 0.001, compared with the SCII+si-NC group; ^###^*P* < 0.001, compared with the SCII+si-HOTAIR group.

**Figure 5:** HOTAIR inhibition promoted recovery of spinal cord function in rats with SIC by modulating the HMGB1/ROS/NF-*κ*B signaling pathway. (a) ROS staining assay. (b) Western blot assay for p65/p-p65 and I-*κ*B*α*/p-I-*κ*B*α* protein levels. ^∗∗∗^*P* < 0.001, compared with the SCII+si-NC group; ^###^*P* < 0.001, compared with the SCII+si-HOTAIR group; ^@@@^*P* < 0.001, compared with the SCII+si-HOTAIR+HMGB1 group.

## Data Availability

No data were used to support this study.
